RETRACTED

# A novel observation of pubic osteomyelitis due to *Streptococcus viridans *after dental extraction: a case report

**DOI:** 10.1186/1752-1947-2-255

**Published:** 2008-07-31

**Authors:** Naseem Naqvi, Rizwana Naqvi, Christopher Wong, Sushmita Pearce

**Affiliations:** 1 Department of Acute Medicine, Dumfries & Galloway Royal Infirmary, UK; 2 Department of Medicine, Macclesfield District General Hospital, East Cheshire NHS Trust, UK; 3 Department of Renal Medicine, Aintree University Hospitals NHS Trust, Liverpool, UK; 4 Department of Medicine, Royal Albert Edward Infirmary, Wigan, UK

## Abstract

**Introduction:**

Pubic osteomyelitis should be suspected in athletic individuals with sudden groin pain, painful restriction of hip movements and fever. It is an infrequent and confusing disorder, which is often heralded by atypical gait disturbance and diffuse pain in the pelvic girdle. The most common pathogen is *Staphylococcus aureus *but, on occasions, efforts to identify infectious agents sometimes prove negative. Pubic osteomyelitis due to *Streptococcus viridans *has not been reported previously in the literature.

**Case presentation:**

We describe the case of a fit 24-year-old athlete, who had a wisdom tooth extracted 2 weeks prior to the presentation, which could have served as a port of entry and predisposed the patient to transient bacteraemia.

**Conclusion:**

*S. viridans *is well known for causing infective endocarditis of native damaged heart valves, but to the best of the authors' knowledge it has not been reported previously as a cause of pubic osteomyelitis. We believe that this case should alert physicians to the association between dental procedures and osteomyelitis of the pubis secondary to *S. viridans*.

## Introduction

Pubic osteomyelitis is an uncommon osseous infection. It accounts for 2% of all osteomyelitis of bone [1,2]. Groups at risk include intravenous drug users [3], people with diabetes and patients who have undergone urological and/or obstetrical procedures [4]. Another, less well-known predisposing factor is strenuous physical activity in athletes [1]. The most common pathogen causing pubic osteomyelitis is *Staphylococcus aureus*. We describe the case of a patient with pubic osteomyelitis due to *Streptococcus viridans*, which developed after dental extraction.

## Case presentation

A 24-year-old, previously fit and well, male fitness instructor and football player presented to the emergency department complaining of pain in his groin and buttocks. Symptoms started 3 days before he presented to the hospital, and he had engaged in strenuous exercise and jogging for 7 hours the day before admission to the hospital. He thought initially that he had sprained his groin muscles while exercising and decided to defer coming to the hospital. There was no other significant past medical history of any illnesses, although the patient reported having had an extraction of a wisdom tooth 2 weeks prior to this presentation.

RETRACTED

On examination in the emergency department, he was a fit-looking man who appeared very anxious. He was brought into the emergency department in a wheelchair. On initial assessment in the emergency department, he was pyrexial with a temperature of 38.6°C, blood pressure 127/77 mmHg, and a regular pulse of 73 beats per minute. On examination of his musculoskeletal system, he was unable to stand and required the support of two people. Examination of the lower limbs revealed painful restriction of hip flexion and extension, with a power of 5/5 in both hips and knees. There was no overlying erythema or tenderness over the hip joints. On neurological examination, sensations were intact to all modalities (intact light touch, pinprick, joint position and vibration sense) with a flexor plantar response. There were no cranial nerve palsies and the cerebellar examination did not reveal any ataxias or nystagmus. No abnormalities were detected on cardiovascular, respiratory and abdominal examination, apart from mild tenderness in the lower abdomen without guarding or rebound. Bowel sounds were present and genital examination was unremarkable with good anal tone. No tenderness was elicited on examination of the spine.

Initial investigations revealed a normal full blood count (haemoglobin 15.2 g/litre, white blood cell count 8.7 × 10^9^/litre with a neutrophil count of 6.8 × 10^9^/litre and platelets of 412 × 10^9^/litre), normal urea, creatinine and electrolytes with the exception of raised C-reactive protein (CRP) at 142 mg/litre. He was admitted to the acute assessment ward with the possible differential diagnosis of acute myositis or pelvic and/or psoas abscess, and blood cultures were performed. An urgent computed tomography (CT) scan of his abdomen and pelvis did not reveal any evidence of psoas or pelvic abscess and serum creatinine kinase levels were 40 U/litre. Other enzymes including lactate dehydrogenase, aldolase, aspartate transaminase and alanine transaminase were all within normal limits.

On the second day of admission, he started having swinging pyrexia (body temperature spiking to 39°C and touching the baseline of 36.6°C every 6 hours) with rigors. At that time, his weakness and pain were severe enough to limit even turning and sitting up in bed. Repeat examination revealed severe tenderness to palpation over the symphysis pubis, more marked on the left. Initial sets of blood cultures revealed heavy growth of *S. viridans*. He was commenced on high doses of ceftriaxone (2 g three times a day) and gentamicin (80 mg once a day). A magnetic resonance imaging (MRI) scan of the pelvis suggested marrow oedema of the left pubic bone extending all the way up to the left sacro-iliac joint and soft tissue swelling of the pubic symphysis, changes highly suggestive of osteomyelitis of the left pubic ramus (Figure 1).

RETRACTED

**Figure 1:** **Magnetic resonance imaging scan of the pelvis showing extensive marrow oedema of the left pubic ramus**.

A bone scan showed increased uptake of contrast over the left pubic ramus and subsequent needle aspiration of the left pubic bone grew *S. viridans *on cultures. Further investigations to exclude any potential cause of immunodeficiency, including human immunodeficiency virus testing, were negative.

The patient gradually improved on intravenous antibiotics, started ambulating and became apyrexial after a week's course of antibiotics. The level of CRP came down to 50 mg/litre from an initial value of 142 mg/litre. He was later discharged from the hospital on 4 weeks of oral clindamycin. He was reviewed in the clinic 4 weeks after his discharge and showed complete clinical recovery. The CRP level had returned to normal (less than 5 mg/litre) and subsequent blood cultures were sterile.

## Discussion

Pubic osteomyelitis should be suspected in athletic individuals with sudden abdominal, pelvic or groin pain, painful restriction of hip movements and fever. The pathogenesis of this disease in athletes is thought to involve pre-existing trauma or sports injury and subsequent seeding of this area during transient bacteraemia following surgical procedures, for example, dental extraction [4]. The main differential diagnosis of pubic osteomyelitis is osteitis pubis.

Osteitis pubis is a painful, noninfectious, self-limited inflammatory condition of the pubic bone associated mainly with genitourinary surgery, but it also occurs following minor trauma or as a manifestation of overuse in athletes [5]. Whereas the initial clinical symptoms of the two conditions may be similar, the presence of fever and progressive clinical deterioration favours an infectious process and emphasises the need for repeated cultures. It is still unclear why athletes are at risk of developing this rare condition. This condition commonly occurs in specific athletic endeavours, such as football or running, that involve strenuous physical exercise and may produce excessive stress to the pelvis. In addition, it has been suggested that the immune system in athletes may be compromised during strenuous exercise, which might increase their susceptibility to transient bacteraemia caused by minor skin or mucous membrane trauma; however, this issue is debatable. Finally, a pre-existing subclinical osteitis pubis may make athletes locally susceptible to osteomyelitis [5]. It is important to recognise that both conditions may occur simultaneously in one patient [6].

RETRACTED

Osteomyelitis of the pubic bone is an infrequent and confusing disorder, which is often heralded by atypical gait disturbance and diffuse pain in the pelvic girdle [7]. Diagnosis of pubic osteomyelitis is often delayed in young patients as it occasionally mimics pelvic pathology resulting in unnecessary invasive procedures in the search for the cause of an acute onset of lower abdominal pain. Symptoms of fever, nausea, vomiting, anorexia and lower abdominal pain and tenderness in a young patient can easily be mistaken for those of acute appendicitis. The classic symptoms of pubic osteomyelitis include pain in the groin or adjacent areas with radiation to the thigh and limitation of motion. The classic signs include local tenderness and swelling, a high temperature, occasionally an elevated erythrocyte sedimentation rate and leucocytosis. The port of entry of infection is often unclear and any history of preceding injuries, infections or dental procedures should be specifically looked for when eliciting history. Any history of painful restriction of hip movements should be specifically explored as it is often wrongly diagnosed as true muscular weakness of the pelvic girdle muscles or septic arthritis of the hip joint.

We found 19 reported cases of pubic osteomyelitis in athletes, including our patient, in a review of the literature [8]. All patients were active athletes who participated in strenuous physical activity. In most of the 18 other patients, diagnosis was delayed. The average time from the start of symptoms to diagnosis was 13 days (range 1 to 30 days). Changes in plain radiographs of the pubic bone usually appear only several weeks after the clinical presentation of osteomyelitis and, therefore, are not reliable in making the diagnosis. Typical changes include pubic rarefaction and osteolysis. Sclerosis may appear later. A technetium bone scan shows increased uptake and may facilitate an earlier diagnosis. In three patients, diagnosis was made only after aspiration and culture. In most of the cases reviewed, the infectious agent was identified. The most common pathogen was *Staphylococcus aureus*, which was identified in cultures of blood or local aspirate [9]

To the authors' knowledge, *S. viridans *has not been previously reported as a cause of pubic osteomyelitis, although there are case reports of vertebral osteomyelitis caused by *S. viridans *in people with diabetes [10,11] and two cases of femoral osteomyelitis due to *S. viridans *[12,13]. *S. viridans *are aerobic, Gram-positive cocci most abundant in oral flora as commensals and are well known for causing infective endocarditis of native damaged heart valves although, in our patient, there was no clinical evidence of endocarditis as evidenced by a normal transoesophageal echocardiogram. Dental extraction in our patient could have served as a port of entry and predisposed the patient to transient bacteraemia.

RETRACTED

## Conclusion

Pubic osteomyelitis is a challenging diagnostic dilemma. We believe that this novel observation should alert physicians to the association between dental procedures and pubic osteomyelitis due to *S. viridans*. It is important to take a history of dental extraction in all patients who present with fever and pelvic pain. It is also important to investigate patients with MRI scans as X-rays are neither sensitive nor specific enough for detecting osteomyelitis. Changes in plain radiographs of the pubic bone usually appear only several weeks after the clinical presentation of osteomyelitis and therefore are not reliable in making the diagnosis. Early diagnosis and treatment can prevent subsequent deformities of the pelvic bones and morbidity due to chronic osteomyelitis and joint deformities.

## Competing interests

The authors declare that they have no competing interests.

## Authors' contributions

NN Chief author, RN Assisted in the preparation of manuscript, SP Consultant in-charge for the patient's management, as well as ideas for the writing of the case report, CW Proof-read the manuscript.

## Consent

Written informed consent was obtained from the patient for publication of this case report and any accompanying images. A copy of the written consent is available for review by the Editor-in-Chief of this journal.
